# Monitoring Mortality Caused by COVID-19 Using Gamma-Distributed Variables Based on Generalized Multiple Dependent State Sampling

**DOI:** 10.1155/2021/6634887

**Published:** 2021-04-22

**Authors:** Muhammad Aslam, G. Srinivasa Rao, Muhammad Saleem, Rehan Ahmad Khan Sherwani, Chi-Hyuck Jun

**Affiliations:** ^1^Department of Statistics, Faculty of Science, King Abdulaziz University, Jeddah 21551, Saudi Arabia; ^2^Department of Mathematics and Statistics, CNMS, The University of Dodoma, Dodoma, PO Box: 259, Tanzania; ^3^Department of Industrial Engineering, Faculty of Engineering-Rabigh, King Abdulaziz University, Jeddah 21589, Saudi Arabia; ^4^College of Statistical and Actuarial Sciences, University of the Punjab Lahore, Pakistan; ^5^Department of Industrial and Management Engineering, POSTECH, Pohang 790-784, Republic of Korea

## Abstract

More recently in statistical quality control studies, researchers are paying more attention to quality characteristics having nonnormal distributions. In the present article, a generalized multiple dependent state (GMDS) sampling control chart is proposed based on the transformation of gamma quality characteristics into a normal distribution. The parameters for the proposed control charts are obtained using in-control average run length (ARL) at specified shape parametric values for different specified average run lengths. The out-of-control ARL of the proposed gamma control chart using GMDS sampling is explored using simulation for various shift size changes in scale parameters to study the performance of the control chart. The proposed gamma control chart performs better than the existing multiple dependent state sampling (MDS) based on gamma distribution and traditional Shewhart control charts in terms of average run lengths. A case study with real-life data from ICU intake to death caused by COVID-19 has been incorporated for the realistic handling of the proposed control chart design.

## 1. Introduction

One of the important techniques for improving manufactured product quality and for reducing the manufacturing costs is statistical quality control (SQC). Since the pioneer work by Shewhart A. Walter during 1920s in Bell Telephone Laboratories, wide varieties of control chart techniques have been constructed and extensively implemented in SQC. The main feature of control charting is to identify the amount of assignable cause(s) and hence rectify it by taking necessary action on the production process before sending the outcome of the products into the market. This control charting helps to avoid nonconforming products from being manufactured by the company. More details about Shewhart control charts can be seen in Montgomery [1].

Usually, control charts are being designed and operating under the assumption of the normality for the variable of interest. Nevertheless, these assumptions may not be true for various realistic situations and other distributions away from normality had been considered and discussed by many authors in the literature (e.g., see [2–5]). The waiting time of an event, for example, can be represented by a gamma distribution as in [6]. Numerous researchers concentrate on quality characteristic understudy which follows a nonnormal distribution or transformed into normality to apply Shewhart type control charts. For skewed data, the gamma distribution is widely used. The works on the control charts for the gamma distribution are presented by Al-Oraini and Rahim [7], Jearkpaporn et al. [8], Sheu and Lin [9], Aslam et al. [10], and Zhang et al. [11]. Santiago and Smith [5] used transformation given by Johnson and Kotz [12] and Nelson [13]. Mohammed [14], Mohammed and Laney [15], and Aslam et al. [16] discussed the application of the *t*-chart.

Several researchers have developed diversified sampling designs to obtain more efficient control charts. Recently, researchers focused on multiple dependent state (MDS) sampling in the creation of a control chart. Wortham and Baker [17] proposed the MDS sampling in quality control charts. MDS design is more competent than the existing single sampling plans because it considers the previous lot information along with the current lot to make a decision whether the process is under control or not (see [18]). Aslam et al. [19] developed a control chart for gamma distribution using MDS sampling. The control chart scheme using MDS sampling was studied by different authors for various schemes (see [16, 19, 20–29, 30, 31]).

More recently, Raza and Aslam [32], Rao et al. [33], Rao et al. [34], and Aslam et al. [35, 36] formulated generalized MDS (GMDS) sampling for various schemes. GMDS is more flexible and efficient than MDS to design the control chart using the gamma distribution. The aim of this article is to construct a gamma control chart for monitoring the process mean based on GMDS sampling design. The application of the proposed chart will be given using the COVID-19 mortality data. It is expected that the proposed chart will perform better than the existing Shewhart control chart and control charts using MDS in terms of average run length and standard deviation of run length.

## 2. Design of Control Chart for Gamma Distribution Based on GMDS Sampling

The proposed control chart for a gamma distribution using gamma to normal transformation is discussed. Let *X* be a random variable from a gamma distribution with shape parameter *α* and scale parameter *β*. The cumulative distribution function (cdf) of the gamma distribution is given by

(1) $$\begin{array}{c} p\left(X\leq x\right)=1-\overset{\alpha -1}{\underset{k=0}{\sum }}\frac{e^{-x/\beta }{\left(x/\beta \right)}^{k}}{k!}. \end{array}$$

Wilson and Hilferty [37] recommended that if *X* follows a gamma distribution with specific parameters, then the transformed variable *X*^∗^ = *X*^1/3^ can be distributed approximately as normal with mean *μ*_*X*^∗^_ and variance *σ*_*X*^∗^_^2^, where

(2) $$\begin{array}{c} \mu_{X^{*}}=\frac{\beta^{1/3}\Gamma \left(\alpha +1/3\right)}{\Gamma \alpha },\\ \sigma_{X^{*}}^{2}=\frac{\beta^{2/3}\Gamma \left(\alpha +2/3\right)}{\Gamma \alpha }-\mu_{X^{*}}^{2}. \end{array}$$

The proposed gamma control chart using GMDS sampling comprises the two pairs of control chart limits. The inner lower control limit (LCL) and upper control limit (UCL) are denoted by subscript 1, and the outer lower control limit (LCL) and upper control limit (UCL) are denoted by subscript 2. The four control limits are given by

(3) $$\begin{array}{c} {\text{UCL}}_{1}=\mu_{X^{*}}+k_{1}\sigma_{X^{*}}=\frac{\beta^{1/3}\Gamma \left(\alpha +1/3\right)}{\Gamma \alpha }+k_{1}\sqrt{\frac{\beta^{2/3}\Gamma \left(\alpha +2/3\right)}{\Gamma \alpha }-\mu_{X^{*}}^{2}}, \end{array}$$

(4) $$\begin{array}{c} {\text{LCL}}_{1}=\mu_{X^{*}}-k_{1}\;\sigma_{X^{*}}=\frac{\beta^{1/3}\Gamma \left(\alpha +1/3\right)}{\Gamma \alpha }-k_{1}\sqrt{\frac{\beta^{2/3}\Gamma \left(\alpha +2/3\right)}{\Gamma \alpha }-\mu_{X^{*}}^{2}}, \end{array}$$

(5) $$\begin{array}{c} {\text{UCL}}_{2}=\mu_{X^{*}}+k_{2}\sigma_{X^{*}}=\frac{\beta^{1/3}\Gamma \left(\alpha +1/3\right)}{\Gamma \alpha }+k_{2}\sqrt{\frac{\beta^{2/3}\Gamma \left(\alpha +2/3\right)}{\Gamma \alpha }-\mu_{X^{*}}^{2}}, \end{array}$$

(6) $$\begin{array}{c} {\text{LCL}}_{2}=\mu_{X^{*}}-k_{2}\sigma_{X^{*}}=\frac{\beta^{1/3}\Gamma \left(\alpha +1/3\right)}{\Gamma \alpha }-k_{2}\sqrt{\frac{\beta^{2/3}\Gamma \left(\alpha +2/3\right)}{\Gamma \alpha }-\mu_{X^{*}}^{2}}, \end{array}$$

where *k*_1_ and *k*_2_ are the chart constants to be found when the in-control ARL is approximately equal to preassigned value *r*_0_. The convenient form of the above control limits is given as follows: UCL_1_ = *β*^1/3^UL_1_, UCL_2_ = *β*^1/3^UL_2_, LCL_1_ = *β*^1/3^LL_1_, and LCL_2_ = *β*^1/3^LL_2_, where

(7) $$\begin{array}{c} {\text{LL}}_{1}=\frac{\Gamma \left(\alpha +1/3\right)}{\Gamma \alpha }-k_{1}\sqrt{\frac{\Gamma \left(\alpha +2/3\right)}{\Gamma \alpha }-{\left(\frac{\Gamma \left(\alpha +1/3\right)}{\Gamma \alpha }\right)}^{2}}, \end{array}$$

(8) $$\begin{array}{c} {\text{LL}}_{2}=\frac{\Gamma \left(\alpha +1/3\right)}{\Gamma \alpha }-k_{2}\sqrt{\frac{\Gamma \left(\alpha +2/3\right)}{\Gamma \alpha }-{\left(\frac{\Gamma \left(\alpha +1/3\right)}{\Gamma \alpha }\right)}^{2}}, \end{array}$$

(9) $$\begin{array}{c} {\text{UL}}_{1}=\frac{\Gamma \left(\alpha +1/3\right)}{\Gamma \alpha }+k_{1}\sqrt{\frac{\Gamma \left(\alpha +2/3\right)}{\Gamma \alpha }-{\left(\frac{\Gamma \left(\alpha +1/3\right)}{\Gamma \alpha }\right)}^{2}}, \end{array}$$

(10) $$\begin{array}{c} {\text{UL}}_{2}=\frac{\Gamma \left(\alpha +1/3\right)}{\Gamma \alpha }+k_{2}\sqrt{\frac{\Gamma \left(\alpha +2/3\right)}{\Gamma \alpha }-{\left(\frac{\Gamma \left(\alpha +1/3\right)}{\Gamma \alpha }\right)}^{2}}. \end{array}$$

The operation of the proposed control chart using GMDS scheme is described as follows:

1. Obtain quality measurement from the manufacturing process, and denote the quality characteristic by *X*. Compute the transformed variable *X*^∗^ as *X*^∗^ = *X*^1/3^
2. The process can be considered under control if LCL_2_ ≤ *X*^∗^ ≤ UCL_2_, and the process can be considered out-of-control if *X*^∗^ ≥ UCL_1_ or *X*^∗^ ≤ LCL_1_. Or else, go to Step 3
3. The process can be considered under control whenever *k* out of *m* proceeding subgroups have been declared as under control, that is, LCL_2_ ≤ *X*^∗^ ≤ UCL_2_; otherwise, the output of the product can be considered out-of-control and go back to Step 1

The probability of declaring as in-control for the proposed control chart when the process is actually in-control is given as follows:

(11) $$\begin{array}{c} P_{\text{in}.0}=P_{a.0}+P_{s.0}\left[\overset{m}{\underset{j=k}{\sum }}\left(\begin{array}{c} m\\ j \end{array}\right)P_{a.0}^{j}{\left(1-P_{a.0}\right)}^{m-j}\right], \end{array}$$

where

(12) $$\begin{array}{c} P_{a.0}=p\left({\text{LCL}}_{2}\leq X^{*}\leq {\text{UCL}}_{2}\;|\;\beta =\beta_{0}\right)=p\left(X^{*}\leq {\text{UCL}}_{2}\;|\;\beta =\beta_{0}\right)-p\left(X^{*}\leq {\text{LCL}}_{2}\;|\;\beta =\beta_{0}\right)=\overset{\alpha -1}{\underset{k=0}{\sum }}\frac{e^{-{\text{LL}}_{2}^{3}}{\left({\text{LL}}_{2}^{3}\right)}^{k}}{k!}-\overset{\alpha -1}{\underset{k=0}{\sum }}\frac{e^{-{\text{UL}}_{2}^{3}}{\left({\text{UL}}_{2}^{3}\right)}^{k}}{k!}, \end{array}$$

(13) $$\begin{array}{c} P_{s.0}=p\left({\text{LCL}}_{1}\leq X^{*}\leq {\text{LCL}}_{2}\;|\;\beta =\beta_{0}\right)+p\left({\text{UCL}}_{2}\leq X^{*}\leq {\text{UCL}}_{1}\;|\;\beta =\beta_{0}\right)=\overset{\alpha -1}{\underset{k=0}{\sum }}\frac{e^{-{\text{LL}}_{1}^{3}}{\left({\text{LL}}_{1}^{3}\right)}^{k}}{k!}-\overset{\alpha -1}{\underset{k=0}{\sum }}\frac{e^{-{\text{LL}}_{2}^{3}}{\left({\text{LL}}_{2}^{3}\right)}^{k}}{k!}+\overset{\alpha -1}{\underset{k=0}{\sum }}\frac{e^{-{\text{UL}}_{2}^{3}}{\left({\text{UL}}_{2}^{3}\right)}^{k}}{k!}-\overset{\alpha -1}{\underset{k=0}{\sum }}\frac{e^{-{\text{UL}}_{1}^{3}}{\left({\text{UL}}_{1}^{3}\right)}^{k}}{k!}. \end{array}$$

Therefore, the in-control average run length (ARL) when the process is under control is given by

(14) $$\begin{array}{c} {\text{ARL}}_{0}=\frac{1}{1-P_{\text{in}.0}}. \end{array}$$

Assume the gamma scale parameter has been changed from *β* = *β*_0_ to *β* = *β*_1_ = *sβ*_0_, where *s* is the shift value.

The probability of process is declared as in-control while the scale parameter which has been changed can be obtained as follows:

(15) $$\begin{array}{c} P_{\text{in}.1}=P_{a.1}+P_{s.1}\left[\overset{m}{\underset{j=k}{\sum }}\left(\begin{array}{c} m\\ j \end{array}\right)P_{a.1}^{j}{\left(1-P_{a.1}\right)}^{m-j}\right], \end{array}$$

where

(16) $$\begin{array}{c} P_{a.1}=p\left({\text{LCL}}_{2}\leq X^{*}\leq {\text{UCL}}_{2}\;|\;\beta =\beta_{1}\right)=p\left(X^{*}\leq {\text{UCL}}_{2}\;|\;\beta =\beta_{1}\right)-p\left(X^{*}\leq {\text{LCL}}_{2}\;|\;\beta =\beta_{1}\right)=\overset{\alpha -1}{\underset{k=0}{\sum }}\frac{e^{-{\text{LL}}_{2}^{3}/s}{\left({\text{LL}}_{2}^{3}/s\right)}^{k}}{k!}-\overset{\alpha -1}{\underset{k=0}{\sum }}\frac{e^{-{\text{UL}}_{2}^{3}/s}{\left({\text{UL}}_{2}^{3}/s\right)}^{k}}{k!}, \end{array}$$

(17) $$\begin{array}{c} P_{s.1}=p\left({\text{LCL}}_{1}\leq X^{*}\leq {\text{LCL}}_{2}\;|\;\beta =\beta_{1}\right)+p\left({\text{UCL}}_{2}\leq X^{*}\leq {\text{UCL}}_{1}\;|\;\beta =\beta_{1}\right)=\overset{\alpha -1}{\underset{k=0}{\sum }}\frac{e^{-{\text{LL}}_{1}^{3}/s}{\left({\text{LL}}_{1}^{3}/s\right)}^{k}}{k!}-\overset{\alpha -1}{\underset{k=0}{\sum }}\frac{e^{-{\text{LL}}_{2}^{3}/s}{\left({\text{LL}}_{2}^{3}/s\right)}^{k}}{k!}+\overset{\alpha -1}{\underset{k=0}{\sum }}\frac{e^{-{\text{UL}}_{2}^{3}/s}{\left({\text{UL}}_{2}^{3}/s\right)}^{k}}{k!}-\overset{\alpha -1}{\underset{k=0}{\sum }}\frac{e^{-{\text{UL}}_{1}^{3}/s}{\left({\text{UL}}_{1}^{3}/s\right)}^{k}}{k!}. \end{array}$$

The out-of-control average run length (ARL) when the process is out-of-control is given as

(18) $$\begin{array}{c} {\text{ARL}}_{1}=\frac{1}{1-P_{\text{in}.1}}. \end{array}$$

The proposed control chart parameters *k*_1_ and *k*_2_ along with ARL_1_ are obtained using the following algorithm:

1. Decide the predetermined in-control ARL as *r*_0_
2. Fix the known values for *m* and *k*
3. Obtain the ARL_0_ using Equation (14), which consists of chart parameters *k*_1_ and *k*_2_
4. Determine the most possible values of chart parameters *k*_1_ and *k*_2_ such that, ARL_0_ ≥ *r*_0_
5. In the above step, we get more values of *k*_1_ and *k*_2_ to satisfy the condition. Choose the best values of *k*_1_ and *k*_2_ for which the value of ARL_0_ is almost equal to *r*_0_
6. Using the best parametric values of *k*_1_ and *k*_2_ determined in the previous step, work out the ARL_1_ using Equation (18) and hence obtain standard deviation (SD) of run-length (SDRL) for various shift (*s*) values

The R codes to find the design parameters of the control chart are given in the appendix.

## 3. Numerical Results and Discussion

The performance of the proposed gamma control chart using GMDS sampling is considered based on ARL, such as ARL_0_ and ARL_1_. These ARL values are used to know the effectiveness of the developed control chart. The developed chart is said to be efficient if it shows larger in-control ARL and smaller out-of-control ARL. Using the aforementioned algorithm in Section 2, the chart coefficients *k*_1_ and *k*_2_ are obtained. The out-of-control ARLs and SDRL are computed for a choice of shift values, *s* from 1.0 to 2.0 with an interval of 0.1 and 2.0 to 4.0 with an interval of 0.5. The values of *m* considered are 4, 5, and 6 and *α*_0_ = 5, 10, and 20.  Table 1 is for *r*_0_ = 370 and *α*_0_ = 5, Table 2 is for *r*_0_ = 370 and *α*_0_ = 10, Table 3 is for *r*_0_ = 370 and *α*_0_ = 20, Table 4 is for *r*_0_ = 500 and *α*_0_ = 5, Table 5 is for *r*_0_ = 500 and *α*_0_ = 10, and Table 6 is for *r*_0_ = 500 and *α*_0_ = 20.

We pointed out the following several noteworthy comments from Tables 1–6 for the developed control charts:

1. The out-of-control ARL and SDRL values decline speedily when the shift (*s*) of the manufacturing process increases
2. It is detected that the chart coefficient *k*_2_ shows an increasing tendency for increased value of *k* for a fixed value of *m* when other parametric combinations are fixed
3. From the tables, it is noticed that ARL_1_ and SDRL values decrease when *m* values increase. In addition, ARL_1_ and SDRL values increased with the increase of *k* value (i.e., *m*-2 to *m*-0). It also observed the same inclination over the other parametric combinations and ARL_0_ = 370 and 500
4. It is interesting to observe from the results that the values of ARL_1_ and SDRL are small for *k* = *m*-2 and these values are increasing from *k* = *m*-2 to *k* = *m* for fixed values of *m*. In addition, noticed that ARL_1_ and SDRL values are large at *k* = *m* as compared to the values at *k* = *m*-1 and *k* = *m*-2 (we know that if *k* = *m*, the developed plan becomes MDS design). Hence, it is concluded from the results that gamma control chart using GMDS sampling is an enormous amount of accurate than gamma control chart using MDS sampling

## 4. Comparison with Existing Charts

In this part, a comparison is made between the developed control chart and the existing Shewhart type control chat and MDS control chart for gamma distribution. Also, the application of developed control chart and its dominance over available control chart schemes studied using real data set is presented. In addition, through a simulation study, the supremacy of the developed control chart when compared with the existing control charts is examined. The performance of the developed control chart is studied through ARL values and we know that a control chart with smaller ARL values is more desirable. In this investigation, we studied when ARL_0_ = 370 and ARL_0_ = 500; the shape parameter of gamma distribution is given as *α*_0_ = 5, 10, and 20 to compare the developed gamma control chart under GMDS with the existing MDS and Shewhart type control chart at various shift values. These comparisons are presented in Table 7 for ARL_0_ = 370 and *m* = 4 and in Table 8 for ARL_0_ = 500 and *m* = 5 at various shape parameters of the gamma distribution.

It is noticed that from the results on the basis of Tables 7 and 8, the developed gamma control charts show smaller quantity ARL_1_ values as compared with the MDS and Shewhart type control charts at various shifts (*s*) values and various parametric values studied in this article. At a glance, when ARL_0_ = 370, *α*_0_ = 5 and *s* = 1.4 from Table 7, for the developed control chart ARL_1_ = 27.17 whereas ARL_1_ = 31.10 for MDS scheme and ARL_1_ = 38.44 from the Shewhart type control chart. Similarly, for ARL_0_ = 500, *α*_0_ = 10, and *s* = 1.5 from Table 8, we sense that the developed control chart gives ARL_1_ = 5.67 while ARL_1_ = 7.22 for the MDS control chart and ARL_1_ = 14.28 from the Shewhart type control chart. The graphical presentation is given to show the performance of developed control chat over the existing MDS and Shewhart type control charts along with various shift values (see Figures 1 and 2). From these two figures, it is articulated that the developed gamma control chart based on GMDS is certified extra sensitive as compared to the MDS and the Shewhart-type control charts. To draw attention to this conclusion, a real data illustration and a simulation study are also carried out in the following subsections.

### 4.1. Simulation Analysis

In order to investigate the implementation of the planned control chart over the available control charts, a simulation study is conducted. In this investigation, 30 samples are generated from the gamma distribution with shape parameter *α*_0_ = 5 and in-control scale parameter 1 and last 30 random samples are generated from a gamma distribution with shape parameter *α*_0_ = 5 and out-of-control scale parameter 1.4 (i.e., the shift of *s* = 1.4). The data is reported in Table 9 alongside computed statistic *X*_*i*_^∗^ = *X*_*i*_^1/3^. The control chart coefficients at *m* = 5, *α*_0_ = 5, and ARL_0_ = 500 are available in Table 8. The Shewhart type gamma control chart is given in Figure 3, and MDS gamma control chart when *m* = 5 and *k* = 5 is provided in Figure 4. The gamma control chart using GMDS sampling when *m* = 5 and *k* = 3 is depicted in Figure 5. According to the above scheme for gamma control charts, we implement the MDS chart as follows: if previous 5 (since *m* = 5) *X*_*i*_^∗^ values are displayed between the inner control limits, then the process is considered to be under control while for proposed gamma control chart under GMDS, the process is said to be declared as under control if no less than 3 out of 5 previous (since *k* = 3 and *m* = 5) *X*_*i*_^∗^ values are within the interior control limits.

From Figures 3 and 4, it is apparent that the gamma control charts based on Shewhart type and MDS scheme are unable to notice the shift. On the other hand, in Figure 5, it can be found that using gamma control charts under the GMDS scheme detects out-of-control at sample numbers 34, 40, 41, 44, 45, 50, and 59. Present simulation examines that the developed gamma control chart based on GMDS sampling is more efficient than the gamma control charts as compared to MDS and Shewhart type design.

### 4.2. Application of the Proposed Chart for COVID-19 Data

In the present section, the developed gamma control chart using GMDS sampling is applied to the monitoring of Coronavirus (COVID-19) outbreak in China. The data set is borrowed from Li et al. [38], and they discussed mortality caused by COVID-19 based on collected data of 33 death cases in Wuhan city of Hubei province during an early outbreak as well as confirmed cases and death toll. They have studied the COVID-19 outbreak in China by considering some specific regions as representative samples. The days from ICU intake to death caused by COVID-19 data are presented in Table 10 along with the transformation of the variable. To fit the gamma distribution, the parameters are estimated using the maximum likelihood approach, and the shape is 2.0026≈2.0, and the scale parameter is 3.9185. The Kolmogorov-Smirnov test is 0.1197, and *p* value is 0.7322.  Figure 6 displays the histogram and Q-Q plot to highlight the goodness of fit of the gamma distribution. Hence, gamma distribution furnishes a good fit for the days from ICU intake to death caused by COVID-19 data.

The chart constants at the estimated shape parameter of 2 are obtained using a simulation procedure given in Section 2. The control chart constants at *α*_0_ = 2 and *m* = 4 are *k*_1_ = 3.1035 and *k*_2_ = 1.4645 for a developed control chart, *k*_1_ = 3.7525 and *k*_2_ = 2.1935 for MDS control chart, and *L* = 2.8828 for Shewhart type control chart. The chart limits of the developed control chart, MDS, and Shewhart type control charts for days from ICU intake to death data are given in Figures 7–9. In Figures 7–9, the proposed control charts for GMDS, MDS, and Shewhart type control charts are displayed by plotting the control limits and chat statistics*X*^∗^. Using days from ICU intake to death data, the developed control chart can be exemplified as follows: declare the process as in-control when 4 earlier values of *X*^∗^ fall in the inner control limits of the developed gamma control chart using the MDS plan. While in the case of the developed gamma control chart using GMDS scheme, the process can be expected as in-control when at least 2 out of 4 earlier values of *X*^∗^ fall in the inner control limits.

It is clearly noticeable from Figure 7 that all sample statistics are inside the upper and lower control limits. Hence, it shows that Shewhart-type gamma control chart fails to detect a change in the process. On the other hand, if we consider gamma control chart, using MDS design also failed to identify changes in the process due to all sample statistics inside the inner upper and inner lower control limits (see Figure 8), whereas the gamma control chart based on GMDS design experiences the out-of-control signals at sample numbers 10, 13, 23, 31, and 33, respectively (see Figure 9). Therefore, from the methodology explained in Section 2, it reveals that the developed gamma control chart based on GMDS design is faster in detecting process variation as compared with the existing control chart based MDS and Shewhart type. Hence, from real application in the field of medical sciences, data for days from ICU intake to death revels that the gamma control chart based on GMDS remains superior methodology as compared to the existing control charts considered in this study.

## 5. Conclusions

We developed the gamma control chart based on GMDS sampling. The computational methodology is also discussed for ARL and SDRL when the process is in-control and out-of-control. The control chart parameters for the proposed control chart are obtained using in-control average run length (ARL_0_) and out-of-control ARL (ARL_1_) of the proposed gamma control chart using GMDS sampling. The performance of the proposed control chart is investigated using simulation for the various shifts in the scale parameter. Tables of chart parameters alongside out-of-control ARL (ARL_1_) for various shift values for specified shape parameters are displayed. Furthermore, a comparative study is also carried out with the developed gamma control chart based on GMDS sampling over the existing MDS and Shewhart type gamma control charts using the ARLs. The results display that the developed gamma control chart based on GMDS sampling shows reduced ARL_1_ values as compared with the existing two gamma control chart discussed in this article.

The implementation of the developed control chart is demonstrated using simulation study as well as tangible data from ICU intake to death cause by COVID-19 and it is shown that designed gamma control chart using GMDS sampling detected out-of-control samples whereas the MDS and Shewhart type gamma control charts failed to detect the out-of-control signal. Hence, we conclude that the gamma control chart based on GMDS is a superior methodology as compared to the existing control charts considered in this study to detect a shift in the parameter. The developed control chart method in this paper can be used in different industrial and medical situations specifically when the researcher would like to discover a small and moderate shift in quality characteristics. Future research maybe considered as control charts for some nonnormal distributions and cost consideration using GMDS sampling design.

## Figures and Tables

**Figure 1:** ARL curves of gamma control chart for three charts for *m* = 4 and ARL_0_ = 370.

**Figure 2:** ARL curves of gamma control chart for three charts for *m* = 5 and ARL_0_ = 500.

**Figure 3:** Gamma control chart for Shewhart type for simulated data when *m* = 5, *α*_0_ = 5, and ARL_0_ = 500.

**Figure 4:** Gamma control chart using MDS sampling for simulated data when *m* = 5, *α*_0_ = 5, and ARL_0_ = 500.

**Figure 5:** Gamma control chart using GMDS sampling for simulated data when *m* = 5, *α*_0_ = 5, and ARL_0_ = 500.

**Figure 6:** The empirical and theoretical cdfs and Q-Q plots for the GD for the days from ICU intake to death.

**Figure 7:** Shewhart type gamma control chart for days from ICU intake to death data.

**Figure 8:** Gamma control chart using MDS sampling for days from ICU intake to death data.

**Figure 9:** Gamma control chart using GMDS sampling for days from ICU intake to death data.

**Table 1:** ARLs and SDRLs of proposed control chart for gamma distribution when *α*_0_ = 5 and ARL_0_ = 370.

*s*	*k*_1_ = 3.1125		*k*_1_ = 3.0045		*k*_1_ = 3.0025		*k*_1_ = 3.0240		*k*_1_ = 3.0045		*k*_1_ = 3.0060		*k*_1_ = 3.0615		*k*_1_ = 3.0215		*k*_1_ = 3.0225	
	*k*_2_ = 1.5025		*k*_2_ = 2.0305		*k*_2_ = 2.5235		*k*_2_ = 1.6985		*k*_2_ = 2.0955		*k*_2_ = 2.5455		*k*_2_ = 1.7260		*k*_2_ = 2.1075		*k*_2_ = 2.5325	
	*m* = 4, *k* = 2		*m* = 4, *k* = 3		*m* = 4, *k* = 4		*m* = 5, *k* = 3		*m* = 5, *k* = 4		*m* = 5, *k* = 5		*m* = 6, *k* = 4		*m* = 6, *k* = 5		*m* = 6, *k* = 6	
	ARL	SDRL	ARL	SDRL	ARL	SDRL	ARL	SDRL	ARL	SDRL	ARL	SDRL	ARL	SDRL	ARL	SDRL	ARL	SDRL
1.0	370.05	369.55	370.01	369.51	370.02	369.52	370.00	369.50	370.01	369.51	370.04	369.54	370.04	369.54	370.03	369.53	370.02	369.52
1.1	206.61	206.11	207.63	207.13	208.25	207.75	205.73	205.23	206.33	205.83	207.32	206.82	200.51	200.01	203.00	202.50	204.91	204.41
1.2	100.36	99.86	102.57	102.07	104.12	103.62	99.93	99.43	100.88	100.38	103.04	102.54	93.77	93.27	96.97	96.47	100.37	99.87
1.3	50.23	49.73	52.51	52.01	54.56	54.06	49.96	49.45	50.99	50.49	53.68	53.18	45.07	44.56	47.87	47.36	51.62	51.12
1.4	27.17	26.67	29.00	28.50	31.10	30.60	26.86	26.36	27.82	27.31	30.46	29.96	23.48	22.97	25.63	25.13	29.03	28.53
1.5	16.00	15.50	17.37	16.86	19.27	18.77	15.68	15.17	16.49	15.99	18.83	18.33	13.44	12.93	15.04	14.53	17.86	17.35
1.6	10.21	9.70	11.22	10.71	12.87	12.36	9.91	9.40	10.60	10.08	12.56	12.05	8.43	7.92	9.63	9.12	11.91	11.39
1.7	7.00	6.48	7.76	7.24	9.15	8.64	6.74	6.22	7.32	6.80	8.95	8.43	5.75	5.23	6.67	6.15	8.50	7.98
1.8	5.11	4.58	5.69	5.17	6.87	6.35	4.90	4.37	5.38	4.85	6.73	6.21	4.22	3.69	4.94	4.41	6.42	5.90
1.9	3.93	3.39	4.40	3.86	5.39	4.87	3.76	3.22	4.17	3.64	5.31	4.78	3.29	2.74	3.87	3.34	5.09	4.56
2.0	3.16	2.61	3.54	3.00	4.40	3.87	3.03	2.48	3.39	2.84	4.34	3.81	2.69	2.13	3.18	2.63	4.18	3.65
2.5	1.66	1.04	1.86	1.26	2.30	1.73	1.63	1.01	1.84	1.24	2.30	1.73	1.56	0.93	1.80	1.21	2.27	1.70
3.0	1.28	0.60	1.41	0.76	1.67	1.06	1.29	0.61	1.42	0.77	1.68	1.07	1.27	0.59	1.42	0.77	1.67	1.05
3.5	1.14	0.40	1.23	0.54	1.40	0.74	1.16	0.43	1.25	0.55	1.40	0.75	1.16	0.43	1.25	0.56	1.40	0.75
4.0	1.08	0.30	1.15	0.41	1.25	0.56	1.10	0.33	1.16	0.42	1.26	0.57	1.10	0.33	1.16	0.43	1.26	0.57

**Table 2:** ARLs and SDRLs of proposed control chart for gamma distribution when *α*_0_ = 10 and ARL_0_ = 370.

*s*	*k*_1_ = 3.0575		*k*_1_ = 3.0145		*k*_1_ = 3.0135		*k*_1_ = 3.1515		*k*_1_ = 3.0785		*k*_1_ = 3.0765		*k*_1_ = 3.1775		*k*_1_ = 3.1225		*k*_1_ = 3.1145	
	*k*_2_ = 1.5790		*k*_2_ = 2.0750		*k*_2_ = 2.5765		*k*_2_ = 1.6005		*k*_2_ = 2.0085		*k*_2_ = 2.4645		*k*_2_ = 1.6655		*k*_2_ = 2.0190		*k*_2_ = 2.4505	
	*m* = 4, *k* = 2		*m* = 4, *k* = 3		*m* = 4, *k* = 4		*m* = 5, *k* = 3		*m* = 5, *k* = 4		*m* = 5, *k* = 5		*m* = 6, *k* = 4		*m* = 6, *k* = 5		*m* = 6, *k* = 6	
	ARL	SDRL	ARL	SDRL	ARL	SDRL	ARL	SDRL	ARL	SDRL	ARL	SDRL	ARL	SDRL	ARL	SDRL	ARL	SDRL
1.0	370.01	369.51	370.02	369.52	370.02	369.52	370.01	369.51	370.00	369.50	370.05	369.55	370.01	369.51	370.04	369.54	370.01	369.51
1.1	176.21	175.71	178.51	178.01	179.79	179.29	167.40	166.90	168.84	168.33	171.65	171.15	161.99	161.49	163.28	162.77	167.95	167.45
1.2	66.32	65.82	68.99	68.49	71.50	71.00	57.84	57.34	60.02	59.52	64.22	63.71	53.39	52.89	55.46	54.96	61.19	60.69
1.3	27.01	26.51	28.95	28.45	31.61	31.11	21.89	21.38	23.56	23.05	27.11	26.61	19.51	19.00	21.13	20.63	25.42	24.92
1.4	12.65	12.14	13.91	13.40	16.12	15.61	9.89	9.37	10.98	10.47	13.53	13.02	8.70	8.19	9.79	9.28	12.64	12.13
1.5	6.86	6.34	7.67	7.15	9.37	8.85	5.35	4.82	6.08	5.56	7.85	7.33	4.75	4.22	5.48	4.96	7.37	6.85
1.6	4.25	3.72	4.80	4.27	6.08	5.56	3.39	2.84	3.90	3.36	5.16	4.63	3.06	2.52	3.59	3.05	4.90	4.37
1.7	2.94	2.39	3.34	2.80	4.32	3.79	2.43	1.86	2.81	2.26	3.73	3.19	2.25	1.68	2.65	2.09	3.59	3.05
1.8	2.23	1.66	2.54	1.98	3.30	2.75	1.91	1.32	2.21	1.64	2.91	2.36	1.82	1.22	2.13	1.55	2.83	2.27
1.9	1.82	1.22	2.07	1.48	2.66	2.10	1.62	1.00	1.86	1.26	2.40	1.83	1.57	0.94	1.81	1.21	2.35	1.78
2.0	1.56	0.94	1.77	1.16	2.25	1.67	1.43	0.79	1.63	1.02	2.06	1.48	1.41	0.76	1.61	0.99	2.03	1.44
2.5	1.13	0.38	1.22	0.51	1.40	0.75	1.11	0.35	1.19	0.48	1.35	0.68	1.12	0.37	1.20	0.48	1.34	0.68
3.0	1.04	0.20	1.08	0.30	1.16	0.43	1.04	0.20	1.07	0.28	1.14	0.40	1.04	0.21	1.08	0.28	1.14	0.39
3.5	1.02	0.12	1.03	0.19	1.07	0.28	1.02	0.13	1.03	0.18	1.06	0.25	1.02	0.13	1.03	0.18	1.06	0.25
4.0	1.01	0.08	1.02	0.12	1.03	0.18	1.01	0.08	1.01	0.12	1.03	0.17	1.01	0.09	1.01	0.12	1.03	0.17

**Table 3:** ARLs and SDRLs of proposed control chart for gamma distribution when *α*_0_ = 20 and ARL_0_ = 370.

*s*	*k*_1_ = 3.2715		*k*_1_ = 4.1315		*k*_1_ = 4.4505		*k*_1_ = 3.3265		*k*_1_ = 4.5695		*k*_1_ = 4.7925		*k*_1_ = 3.6385		*k*_1_ = 4.6190		*k*_1_ = 4.5345	
	*k*_2_ = 1.4485		*k*_2_ = 1.7555		*k*_2_ = 2.2170		*k*_2_ = 1.5435		*k*_2_ = 1.8270		*k*_2_ = 2.2580		*k*_2_ = 1.5880		*k*_2_ = 1.8835		*k*_2_ = 2.2915	
	*m* = 4, *k* = 2		*m* = 4, *k* = 3		*m* = 4, *k* = 4		*m* = 5, *k* = 3		*m* = 5, *k* = 4		*m* = 5, *k* = 5		*m* = 6, *k* = 4		*m* = 6, *k* = 5		*m* = 6, *k* = 6	
	ARL	SDRL	ARL	SDRL	ARL	SDRL	ARL	SDRL	ARL	SDRL	ARL	SDRL	ARL	SDRL	ARL	SDRL	ARL	SDRL
1.0	370.02	369.52	370.04	369.54	370.05	369.55	370.01	369.51	370.02	369.52	370.05	369.55	370.04	369.54	370.05	369.55	370.05	369.55
1.1	119.55	119.05	120.53	120.02	121.50	120.99	113.23	112.73	114.29	113.79	118.35	117.84	108.88	108.38	109.14	108.64	115.61	115.11
1.2	25.92	25.41	26.74	26.24	29.44	28.93	22.76	22.26	24.26	23.76	28.18	27.67	21.57	21.07	22.44	21.93	27.16	26.65
1.3	7.93	7.41	8.31	7.79	9.94	9.43	7.41	6.90	7.51	7.00	9.54	9.03	6.37	5.85	6.98	6.46	9.24	8.73
1.4	2.90	2.36	3.76	3.22	4.69	4.16	3.31	2.76	3.49	2.94	4.57	4.04	2.94	2.39	3.32	2.78	4.49	3.96
1.5	2.07	1.50	2.27	1.70	2.84	2.29	2.01	1.43	2.17	1.60	2.82	2.26	1.87	1.28	2.13	1.55	2.82	2.26
1.6	1.52	1.00	1.67	1.05	2.05	1.46	1.51	0.88	1.64	1.02	2.05	1.47	1.46	0.82	1.64	1.03	2.07	1.49
1.7	1.33	0.66	1.38	0.73	1.64	1.03	1.28	0.60	1.38	0.73	1.66	1.05	1.27	0.59	1.40	0.75	1.69	1.07
1.8	1.18	0.46	1.23	0.54	1.42	0.77	1.17	0.44	1.24	0.55	1.44	0.79	1.17	0.45	1.26	0.57	1.46	0.81
1.9	1.11	0.34	1.15	0.41	1.28	0.60	1.11	0.34	1.16	0.43	1.30	0.62	1.11	0.35	1.17	0.45	1.31	0.64
2.0	1.06	0.26	1.10	0.33	1.19	0.48	1.07	0.27	1.11	0.34	1.20	0.49	1.07	0.28	1.12	0.36	1.21	0.51
2.5	1.01	0.09	1.01	0.12	1.03	0.18	1.01	0.09	1.02	0.12	1.03	0.19	1.01	0.10	1.02	0.13	1.04	0.19
3.0	1.00	0.03	1.00	0.04	1.01	0.07	1.00	0.03	1.00	0.05	1.01	0.08	1.00	0.04	1.00	0.05	1.01	0.08
3.5	1.00	0.01	1.00	0.02	1.00	0.03	1.00	0.01	1.00	0.02	1.00	0.03	1.00	0.01	1.00	0.02	1.00	0.03
4.0	1.00	0.00	1.00	0.01	1.00	0.01	1.00	0.01	1.00	0.01	1.00	0.01	1.00	0.01	1.00	0.01	1.00	0.01

**Table 4:** ARLs and SDRLs of proposed control chart for gamma distribution when *α*_0_ = 5 and ARL_0_ = 500.

*s*	*k*_1_ = 3.2215		*k*_1_ = 3.7115		*k*_1_ = 4.5980		*k*_1_ = 3.3615		*k*_1_ = 3.9440		*k*_1_ = 4.4575		*k*_1_ = 3.5845		*k*_1_ = 4.3465		*k*_1_ = 4.4760	
	*k*_2_ = 1.5255		*k*_2_ = 1.8115		*k*_2_ = 2.2670		*k*_2_ = 1.5835		*k*_2_ = 1.8755		*k*_2_ = 2.3070		*k*_2_ = 1.6325		*k*_2_ = 1.9275		*k*_2_ = 2.3390	
	*m* = 4, *k* = 2		*m* = 4, *k* = 3		*m* = 4, *k* = 4		*m* = 5, *k* = 3		*m* = 5, *k* = 4		*m* = 5, *k* = 5		*m* = 6, *k* = 4		*m* = 6, *k* = 5		*m* = 6, *k* = 6	
	ARL	SDRL	ARL	SDRL	ARL	SDRL	ARL	SDRL	ARL	SDRL	ARL	SDRL	ARL	SDRL	ARL	SDRL	ARL	SDRL
1.0	500.03	499.53	500.04	499.54	500.05	499.55	500.01	499.51	500.02	499.52	500.05	499.55	500.04	499.54	500.01	499.51	500.05	499.55
1.1	270.28	269.78	271.57	271.07	273.31	272.81	263.92	263.42	266.57	266.07	268.09	267.59	259.99	259.49	262.25	261.75	264.22	263.71
1.2	126.46	125.96	123.19	122.69	126.16	125.66	117.99	117.49	117.61	117.11	121.35	120.84	112.09	111.58	113.21	112.71	117.87	117.37
1.3	61.13	60.63	57.05	56.55	60.15	59.65	54.22	53.72	53.09	52.59	57.08	56.58	49.49	48.99	50.18	49.68	54.94	54.43
1.4	32.08	31.58	28.99	28.48	31.59	31.09	27.29	26.79	26.51	26.00	29.77	29.27	24.18	23.68	24.78	24.28	28.54	28.03
1.5	18.41	17.91	16.37	15.86	18.40	17.89	15.24	14.73	14.84	14.33	17.31	16.80	13.29	12.78	13.82	13.31	16.60	16.09
1.6	11.50	10.99	10.20	9.68	11.75	11.24	9.39	8.88	9.23	8.71	11.09	10.58	8.15	7.63	8.61	8.09	10.67	10.15
1.7	7.74	7.23	6.91	6.39	8.12	7.60	6.31	5.79	6.28	5.75	7.70	7.18	5.49	4.97	5.89	5.37	7.45	6.93
1.8	5.56	5.04	5.02	4.50	5.99	5.46	4.56	4.03	4.60	4.07	5.71	5.19	4.01	3.47	4.35	3.82	5.56	5.04
1.9	4.23	3.69	3.87	3.33	4.65	4.12	3.50	2.96	3.58	3.04	4.48	3.94	3.12	2.57	3.42	2.88	4.39	3.86
2.0	3.36	2.82	3.13	2.58	3.78	3.24	2.83	2.27	2.92	2.37	3.66	3.12	2.56	2.00	2.82	2.27	3.61	3.07
2.5	1.70	1.09	1.69	1.08	2.01	1.42	1.56	0.93	1.66	1.05	2.01	1.42	1.51	0.87	1.66	1.05	2.02	1.44
3.0	1.29	0.62	1.32	0.65	1.51	0.88	1.25	0.56	1.33	0.66	1.52	0.89	1.24	0.55	1.34	0.67	1.54	0.91
3.5	1.15	0.41	1.18	0.46	1.30	0.62	1.14	0.39	1.19	0.48	1.31	0.64	1.14	0.40	1.20	0.49	1.32	0.65
4.0	1.09	0.30	1.11	0.35	1.19	0.48	1.08	0.30	1.12	0.37	1.20	0.49	1.09	0.31	1.13	0.38	1.21	0.50

**Table 5:** ARLs and SDRLs of proposed control chart for gamma distribution when *α*_0_ = 10 and ARL_0_ = 500.

*s*	*k*_1_ = 3.2635		*k*_1_ = 3.8515		*k*_1_ = 4.5495		*k*_1_ = 3.3245		*k*_1_ = 5.0695		*k*_1_ = 4.5285		*k*_1_ = 3.6205		*k*_1_ = 4.4735		*k*_1_ = 4.5660	
	*k*_2_ = 1.5185		*k*_2_ = 1.8085		*k*_2_ = 2.2730		*k*_2_ = 1.6015		*k*_2_ = 1.8730		*k*_2_ = 2.3135		*k*_2_ = 1.6325		*k*_2_ = 1.9290		*k*_2_ = 2.3460	
	*m* = 4, *k* = 2		*m* = 4, *k* = 3		*m* = 4, *k* = 4		*m* = 5, *k* = 3		*m* = 5, *k* = 4		*m* = 5, *k* = 5		*m* = 6, *k* = 4		*m* = 6, *k* = 5		*m* = 6, *k* = 6	
	ARL	SDRL	ARL	SDRL	ARL	SDRL	ARL	SDRL	ARL	SDRL	ARL	SDRL	ARL	SDRL	ARL	SDRL	ARL	SDRL
1.0	500.01	499.51	500.02	499.51	500.05	499.55	500.04	499.54	500.03	499.53	500.05	499.55	500.05	499.55	500.05	499.55	500.05	499.55
1.1	221.13	220.63	222.17	221.66	223.48	222.98	215.54	215.04	217.15	216.65	218.55	218.05	208.30	207.80	209.08	208.58	214.77	214.27
1.2	71.16	70.16	72.21	71.71	75.75	75.25	69.52	69.02	68.15	67.65	72.53	72.03	62.52	62.01	63.20	62.70	70.16	69.66
1.3	25.31	24.81	26.12	25.62	29.11	28.61	24.82	24.32	24.08	23.58	27.61	27.10	21.19	20.68	21.95	21.45	26.55	26.04
1.4	11.06	10.55	11.57	11.06	13.59	13.08	10.76	10.25	10.60	10.09	12.89	12.38	9.05	8.53	9.67	9.16	12.43	11.92
1.5	5.89	5.37	6.21	5.69	7.55	7.03	5.67	5.14	5.73	5.20	7.22	6.70	4.82	4.29	5.29	4.76	7.01	6.49
1.6	3.21	2.88	3.90	3.36	4.82	4.30	3.52	2.98	3.64	3.10	4.66	4.13	3.07	2.53	3.43	2.89	4.58	4.05
1.7	2.50	2.05	2.76	2.21	3.44	2.89	2.49	1.93	2.63	2.07	3.36	2.82	2.24	1.67	2.52	1.96	3.34	2.79
1.8	2.10	1.32	2.15	1.57	2.66	2.10	1.95	1.36	2.08	1.50	2.63	2.07	1.81	1.21	2.03	1.45	2.63	2.07
1.9	1.59	1.15	1.79	1.18	2.19	1.61	1.63	1.02	1.75	1.15	2.18	1.61	1.55	0.93	1.74	1.13	2.20	1.62
2.0	1.44	0.91	1.56	0.94	1.88	1.29	1.44	0.80	1.55	0.92	1.89	1.30	1.40	0.75	1.55	0.93	1.91	1.32
2.5	1.12	0.36	1.15	0.42	1.27	0.59	1.11	0.36	1.16	0.43	1.29	0.61	1.12	0.36	1.17	0.45	1.30	0.62
3.0	1.04	0.20	1.06	0.24	1.11	0.34	1.04	0.20	1.06	0.25	1.11	0.36	1.04	0.21	1.07	0.27	1.12	0.36
3.5	1.01	0.12	1.02	0.15	1.05	0.22	1.02	0.13	1.02	0.16	1.05	0.23	1.02	0.13	1.03	0.17	1.05	0.23
4.0	1.01	0.08	1.01	0.10	1.02	0.15	1.01	0.08	1.01	0.10	1.02	0.15	1.01	0.08	1.01	0.11	1.02	0.15

**Table 6:** ARLs and SDRLs of proposed control chart for gamma distribution when *α*_0_ = 20 and ARL_0_ = 500.

*s*	*k*_1_ = 4.6725		*k*_1_ = 4.2825		*k*_1_ = 4.5495		*k*_1_ = 3.4165		*k*_1_ = 4.4505		*k*_1_ = 4.5120		*k*_1_ = 3.5885		*k*_1_ = 4.6790		*k*_1_ = 4.7185	
	*k*_2_ = 2.2755		*k*_2_ = 1.8025		*k*_2_ = 2.2730		*k*_2_ = 1.5815		*k*_2_ = 1.8740		*k*_2_ = 2.3165		*k*_2_ = 1.6365		*k*_2_ = 1.9295		*k*_2_ = 2.3490	
	*m* = 4, *k* = 2		*m* = 4, *k* = 3		*m* = 4, *k* = 4		*m* = 5, *k* = 3		*m* = 5, *k* = 4		*m* = 5, *k* = 5		*m* = 6, *k* = 4		*m* = 6, *k* = 5		*m* = 6, *k* = 6	
	ARL	SDRL	ARL	SDRL	ARL	SDRL	ARL	SDRL	ARL	SDRL	ARL	SDRL	ARL	SDRL	ARL	SDRL	ARL	SDRL
1.0	500.04	499.54	500.04	499.54	500.05	499.55	500.05	499.55	500.05	499.55	500.05	499.55	500.04	499.54	500.05	499.55	500.05	499.55
1.1	153.53	153.03	154.54	154.04	155.79	155.29	143.46	142.96	145.72	145.22	151.15	150.65	138.53	138.03	139.18	138.68	147.91	147.41
1.2	30.93	30.42	32.11	31.60	35.55	35.05	27.60	27.10	28.87	28.36	33.80	33.30	25.74	25.23	26.67	26.17	32.64	32.13
1.3	8.23	7.72	9.46	8.95	11.44	10.93	8.08	7.06	8.47	7.95	10.89	10.38	7.19	6.67	7.85	7.33	10.55	10.04
1.4	3.29	2.75	4.12	3.58	5.19	4.67	3.58	3.04	3.77	3.23	5.02	4.49	3.17	2.63	3.58	3.04	4.93	4.40
1.5	2.12	1.55	2.41	1.84	3.05	2.51	2.11	1.54	2.29	1.71	3.01	2.46	1.96	1.38	2.24	1.66	3.00	2.45
1.6	1.69	1.08	1.73	1.13	2.15	1.57	1.55	0.93	1.69	1.08	2.15	1.57	1.50	0.87	1.69	1.08	2.17	1.59
1.7	1.36	0.70	1.42	0.77	1.70	1.10	1.31	0.63	1.41	0.76	1.72	1.11	1.29	0.62	1.43	0.78	1.74	1.14
1.8	1.20	0.49	1.25	0.56	1.46	0.81	1.18	0.46	1.26	0.57	1.47	0.84	1.18	0.47	1.28	0.60	1.49	0.86
1.9	1.12	0.36	1.16	0.43	1.31	0.63	1.11	0.36	1.17	0.45	1.32	0.65	1.12	0.37	1.19	0.47	1.33	0.67
2.0	1.07	0.28	1.11	0.34	1.21	0.50	1.07	0.28	1.12	0.36	1.22	0.52	1.08	0.29	1.13	0.38	1.23	0.53
2.5	1.01	0.09	1.01	0.12	1.03	0.19	1.01	0.10	1.02	0.13	1.04	0.20	1.01	0.10	1.02	0.14	1.04	0.20
3.0	1.00	0.03	1.00	0.05	1.01	0.08	1.00	0.04	1.00	0.05	1.01	0.08	1.00	0.04	1.00	0.05	1.01	0.08
3.5	1.00	0.01	1.00	0.02	1.00	0.03	1.00	0.01	1.00	0.02	1.00	0.03	1.00	0.02	1.00	0.02	1.00	0.04
4.0	1.00	0.01	1.00	0.01	1.00	0.01	1.00	0.01	1.00	0.01	1.00	0.02	1.00	0.01	1.00	0.01	1.00	0.02

**Table 7:** Developed gamma control chart ARL comparison with existing control charts when ARL_0_ = 370 and *m* = 4.

*s*	*α*_0_ = 5			*α*_0_ = 10			*α*_0_ = 20		
	Proposed *k*_1_ = 3.1125 *k*_2_ = 1.5025	MDS *k*_1_ = 3.0025 *k*_2_ = 2.5235	Shewhart *L* = 2.9605	Proposed *k*_1_ = 3.0575 *k*_2_ = 1.5790	MDS *k*_1_ = 3.0135 *k*_2_ = 2.5765	Shewhart *L* = 2.9821	Proposed *k*_1_ = 3.2715 *k*_2_ = 1.4485	MDS *k*_1_ = 4.4505 *k*_2_ = 2.2170	Shewhart *L* = 2.9917
1.0	370.05	370.02	370.96	370.01	370.02	370.96	370.02	370.05	370.96
1.1	206.61	208.25	217.16	176.21	179.79	188.41	119.55	121.50	144.07
1.2	100.36	104.12	114.73	66.32	71.50	80.54	25.92	29.44	46.78
1.3	50.23	54.56	63.78	27.01	31.61	38.47	7.93	9.94	19.11
1.4	27.17	31.10	38.44	12.65	16.12	20.97	2.90	4.69	9.59
1.5	16.00	19.27	24.98	6.86	9.37	12.77	2.07	2.84	5.64
1.6	10.21	12.87	17.30	4.25	6.08	8.50	1.52	2.05	3.75
1.7	7.00	9.15	12.64	2.94	4.32	6.07	1.33	1.64	2.73
1.8	5.11	6.87	9.64	2.23	3.30	4.60	1.18	1.42	2.15
1.9	3.93	5.39	7.63	1.82	2.66	3.64	1.11	1.28	1.78
2.0	3.16	4.40	6.22	1.56	2.25	3.00	1.06	1.19	1.55
2.5	1.66	2.30	3.07	1.13	1.40	1.65	1.01	1.03	1.11
3.0	1.28	1.67	2.07	1.04	1.16	1.27	1.00	1.01	1.02
3.5	1.14	1.40	1.63	1.02	1.07	1.12	1.00	1.00	1.00
4.0	1.08	1.25	1.40	1.01	1.03	1.06	1.00	1.00	1.00

**Table 8:** Developed gamma control chart ARLs comparison with existing control charts when ARL_0_ =500 and *m* =5.

*s*	*α*_0_ = 5			*α*_0_ = 10			*α*_0_ = 20		
	Proposed *k*_1_ = 3.3615 *k*_2_ = 1.5835	MDS *k*_1_ = 4.4575 *k*_2_ = 2.3070	Shewhart *L* = 3.0458	Proposed *k*_1_ = 3.3245 *k*_2_ = 1.6015	MDS *k*_1_ = 4.5285 *k*_2_ = 2.3135	Shewhart *L* = 3.0701	Proposed *k*_1_ = 3.4165 *k*_2_ = 1.5815	MDS *k*_1_ = 4.5120 *k*_2_ = 2.3165	Shewhart *L* = 3.0804
1.0	500.01	500.05	500.94	500.04	500.05	500.93	500.05	500.05	500.04
1.1	263.92	268.09	283.07	215.54	218.55	244.74	143.46	151.15	185.05
1.2	117.99	121.35	144.60	69.52	72.53	100.63	27.60	33.80	57.41
1.3	54.22	57.08	78.26	24.82	27.61	46.63	8.08	10.89	22.64
1.4	27.29	29.77	46.15	10.76	12.89	24.79	3.58	5.02	11.04
1.5	15.24	17.31	29.45	5.67	7.22	14.78	2.11	3.01	6.33
1.6	9.39	11.09	20.09	3.52	4.66	9.66	1.55	2.15	4.12
1.7	6.31	7.70	14.47	2.49	3.36	6.80	1.31	1.72	2.96
1.8	4.56	5.71	10.91	1.95	2.63	5.08	1.18	1.47	2.29
1.9	3.50	4.48	8.54	1.63	2.18	3.98	1.11	1.32	1.88
2.0	2.83	3.66	6.90	1.44	1.89	3.24	1.07	1.22	1.61
2.5	1.56	2.01	3.29	1.11	1.29	1.72	1.01	1.04	1.12
3.0	1.25	1.52	2.17	1.04	1.11	1.29	1.00	1.01	1.03
3.5	1.14	1.31	1.69	1.02	1.05	1.14	1.00	1.00	1.01
4.0	1.08	1.20	1.44	1.01	1.02	1.07	1.00	1.00	1.00

**Table 9:** The simulated data when *m* = 5, *α*_0_ = 5, and ARL_0_ = 500.

S. no.	*X*	*X* ^∗^	S. no.	*X*	*X* ^∗^	S. no.	*X*	*X* ^∗^	S. no.	*X*	*X* ^∗^
1	7.6063	1.9666	16	2.3608	1.3315	31	8.0437	2.0036	46	4.6261	1.6662
2	2.8743	1.4218	17	2.5800	1.3715	32	4.6680	1.6713	47	5.4935	1.7645
3	3.2301	1.4782	18	4.9637	1.7058	33	8.6453	2.0524	48	1.9999	1.2599
4	4.6671	1.6712	19	4.1035	1.6010	34	9.1395	2.0908	49	6.4479	1.8613
5	7.0398	1.9165	20	2.7647	1.4035	35	4.0200	1.5900	50	11.1001	2.2307
6	4.3621	1.6339	21	3.8728	1.5704	36	6.2734	1.8443	51	7.4944	1.9569
7	3.5145	1.5204	22	8.0095	2.0008	37	2.7584	1.4024	52	8.1311	2.0109
8	7.8831	1.9902	23	8.3195	2.0263	38	6.4997	1.8662	53	3.4348	1.5088
9	7.2328	1.9339	24	3.2821	1.4861	39	7.6433	1.9698	54	3.2860	1.4867
10	7.0640	1.9187	25	5.5956	1.7753	40	10.1004	2.1616	55	4.8631	1.6942
11	3.7153	1.5488	26	3.4608	1.5126	41	11.0929	2.2302	56	7.6722	1.9723
12	5.0059	1.7106	27	4.2462	1.6193	42	5.9905	1.8162	57	6.2898	1.8459
13	2.6249	1.3794	28	6.6523	1.8807	43	3.9466	1.5803	58	6.1469	1.8318
14	3.6922	1.5456	29	6.5704	1.8730	44	9.1140	2.0888	59	9.3127	2.1039
15	4.5475	1.6567	30	5.2560	1.7387	45	11.0067	2.2244	60	3.2213	1.4769

**Table 10:** Death cause by COVID-19 in Wuhan city of Hubei province in China.

Subgroup no.	Days from ICU intake to death (*X*)	*X* ^∗^	Subgroup no.	Days from ICU intake to death (*X*)	*X* ^∗^
1	4	1.5874	18	17	2.5713
2	6	1.8171	19	5	1.7100
3	5	1.7100	20	8	2.0000
4	7	1.9129	21	8	2.0000
5	5	1.7100	22	8	2.0000
6	4	1.5874	23	1	1.0000
7	2	1.2599	24	12	2.2894
8	6	1.8171	25	10	2.1544
9	10	2.1544	26	12	2.2894
10	1	1.0000	27	4	1.5874
11	7	1.9129	28	4	1.5874
12	9	2.0801	29	2	1.2599
13	22	2.8020	30	4	1.5874
14	11	2.2240	31	1	1.0000
15	6	1.8171	32	11	2.2240
16	8	2.0000	33	25	2.9240
17	14	2.4101			

## Data Availability

The data is given in the paper.

## Appendix

R Coding to Run the Algorithm

## compute mean and standard deviation

mts<-b^(1/3)∗gamma(a+1/3)/gamma(a)

vts<-b^(2/3)∗gamma(a+2/3)/gamma(a)-mts^2

sdts<-sqrt(vts)

## fixing the range of k1 and k2

q1<-seq(2.61,6.96, by =0.0005)

 q2<-seq(1.21,6.86, by =0.0005)

vv<-gamma(a+2/3)/gamma(a)-(gamma(a+1/3)/gamma(a))^2

   ll1<-gamma(a+1/3)/gamma(a)-k1∗sqrt(vv)

   ll2<-gamma(a+1/3)/gamma(a)-k2∗sqrt(vv)

   u1<-gamma(a+1/3)/gamma(a)+k1∗sqrt(vv)

   u2<-gamma(a+1/3)/gamma(a)+k2∗sqrt(vv)

   lcl1<-max(0,b^(1/3)∗ll1)

   ucl1<-b^(1/3)∗ul1

   lcl2<-max(0,b^(1/3)∗ll2)

   ucl2<-b^(1/3)∗ul2

pa<-sum(dpois(0:(a-1),ll2^3))-sum(dpois(0:(a-1),ul2^3))

ps<-sum(dpois(0:(a-1),ll1^3))-sum(dpois(0:(a-1),ll2^3))+sum(dpois(0:(a-1), ul2^3))

      -sum(dpois(0:(a-1),ul1^3))

s1<-pbinom(m, m, pa, lower.tail = TRUE, log.p = FALSE)

      -pbinom(k-1, m, pa, lower.tail = TRUE, log.p = FALSE)

   Pin0<-pa+ps∗s1

   ARL0=1.0/(1.0-Pin0)

   if ((ARL0>=370) && (ARL0<=370.5)) then choose those k1 and k2 values
